The article "To Analyze the Application Value of Perioperative Nursing Care in Patients with Resected Brain Tumor Accompanied with Epileptic Symptoms under Cortical Electrocorticography Monitoring" was published in 2022. Journal: J Healthc Eng.

# To Analyze the Application Value of Perioperative Nursing Care in Patients with Resected Brain Tumor Accompanied with Epileptic Symptoms under Cortical Electrocorticography Monitoring

**DOI:** 10.1155/2022/4012304

**Published:** 2022-01-29

**Authors:** Shouduo Jiang, Chunjing Li, Shanshan Hu, Yan'e Li, Zerong Wang, Ying Bu

**Affiliations:** ^1^Neuroelectrophysiology Room, Yantaishan Hospital, Yantai 264000, China; ^2^Department of Imaging, Zhangqiu District People's Hospital, Jinan 250200, China; ^3^Department of Neurology (I), Affiliated Qingdao Central Hospital, Qingdao University, Qingdao 266042, China; ^4^Department of Internal Medicine, Zhangqiu District People's Hospital, Jinan 250200, China; ^5^Lanzhou University Second Hospital, Lanzhou 730030, China; ^6^Department of Emergency Medical, Zhangqiu District People's Hospital, Jinan 250200, China

## Abstract

**Objective:**

To explore the application value of perioperative nursing for patients with brain tumors with epilepsy symptoms under the cortical electrocorticography (EEG) monitoring.

**Methods:**

A total of 86 patients with brain tumor complicated with epilepsy admitted to the department of brain surgery of our hospital from January 2018 to December 2019 were selected as the research objects, and all underwent resection under cortical EEG monitoring. According to different nursing methods, they were divided into the control group and observation group, each with 43 cases. The control group was given perioperative basic nursing, and the observation group was given perioperative comprehensive nursing. The EEG image of the patient during the operation was observed by a portable EEG monitor. Anxiety and depression were assessed by self-rating anxiety scale (SAS) and self-rating depression scale (SDS) scores. The self-made satisfaction questionnaire was used to investigate the nursing satisfaction. A visual analogue (VAS) score is used to assess pain degree. A multiparameter monitor was used to detect the patient's heart rate (HR), systolic blood pressure (SBP), and diastolic blood pressure (DBP). The quality of life was assessed by the European Organization for Research and Treatment of Cancer Quality of Life Questionnaire-Core 30 (EORTC QLQ-30). The complication rate and recurrence rate were also counted.

**Results:**

Eighty-six patients with epileptic brain tumor developed spikes in 35 cases, including 7 meningiomas, 22 gliomas, and 6 cholesteatomas; 27 cases of sharp waves, including 14 meningiomas, 12 gliomas, and 1 case of cholesteatomas; and 24 cases of complex wave, including 9 cases of meningioma, 13 cases of glioma, and 2 cases of cholesteatoma. There was no significant difference in the scores of SAS, SDS, VAS, HR, SBP, DBP, and quality of life between the two groups at T0. The VAS score increased at T1 and T2, and the increase in the control group was greater than that in the observation group. At T3 and T4, the SAS, SDS, and VAS scores of the two groups decreased, and the observation group decreased more than the control group. HR, SBP, and DBP of the two groups showed an upward trend at T1 and T2, and the increase in the control group was more significant than that in the observation group. At T3, the three indicators of the two groups decreased, and the observation group decreased more significantly than the control group. At T4, the scores of all indicators of the quality of life of the two groups increased, and the observation group increased more significantly than the control group. The nursing satisfaction of the observation group was higher than that of the control group. The complication rate and recurrence rate in the observation group were decreased compared with the control group.

**Conclusion:**

Perioperative comprehensive nursing intervention for patients with epileptic brain tumor undergoing resection under cortical EEG monitoring can reduce or even eliminate the recurrence rate of epilepsy, reduce the patient's pain and stress response, and improve the patient's quality of life. It can also reduce the occurrence of complications, improve nursing satisfaction, thereby improving patient compliance, and has a high clinical application value.

## 1. Introduction

Epilepsy, which has the main clinical characteristic of abnormal discharge of brain neurons, is a relatively common and recurrent transient brain dysfunction syndrome in clinical [1]. The incidence of epilepsy ranks second among all neurological disorders and the second only to stroke [2, 3]. Epilepsy can be caused by cysts, brain malignant tumors, and other reasons, and most of them are secondary diseases. According to reports, the incidence of brain tumors complicated by epilepsy can reach more than 30% [3]. Clinically, surgical resection is mainly used to remove the lesions, but some patients still have symptoms and relapse after surgery, which affects the prognosis [4–6]. In this study, patients with brain tumor accompanied with epilepsy were treated with cortical EEG monitoring resection and different nursing interventions during the perioperative period, aiming to explore the application value of comprehensive nursing in the treatment of patients with brain tumor accompanied with epilepsy by EEG monitoring resection.

## 2. Materials and Methods

### 2.1. The General Information

A total of 86 patients with brain tumor complicated with epilepsy admitted to the brain surgery department of our hospital from January 2018 to December 2019 were selected as the research objects, and all patients underwent cortical EEG monitoring resection. This study was approved by the Ethics Committee of Yantaishan Hospital and the patients. All patients or their families had informed consent and signed an informed consent form. According to different nursing methods, they were divided into the control group and observation group, each with 43 cases. Inclusion criteria were as follows: symptoms such as recurrent vomiting and dizziness, accompanied by decreased vision, weakness of limbs, and increased headaches [7] and epilepsy symptoms including tonic-clonic cramps, sudden loss of consciousness, foaming at the mouth, and urinary incontinence [8]. Exclusion criteria were as follows: severe disorders of the liver, kidney, and other organs and epilepsy induced by other reasons. There was no statistically significant difference between the two groups of general information (*P* > 0.05) (Table 1), and they were comparable.

### 2.2. Methods

#### 2.2.1. Surgical Methods

Both groups underwent resection under the monitoring of cortical EEG intraoperative by the Cadwell Cascade^®^ neurophysiological monitor of the United States. CT scan was performed to determine the location of the lesion, and then, normal tissue (3 cm around the lesion) was exposed to design the location and size of the incision. During craniotomy, a portable EEG monitor was used to record the projection of the lesion site, and the area of suspected epilepsy was detected. The lesion tissue was resected under a microscope, and the flat cortex was scanned with the EEG monitor to remove all the epileptic waves.

#### 2.2.2. Nursing Methods

The control group received basic perioperative care, including providing a comfortable and quiet ward environment, preparing the items needed for the operation, mastering the operation process and performing various cooperation during the operation, and giving dietary guidance and basic precautions after the operation.

On the basis of the control group, the observation group carried out comprehensive nursing intervention. (1) Preoperative care: before the operation, the nurse in the operating room needs to have a comprehensive understanding of the patient's condition, explain the operation method in detail to the patient, communicate with the patient and answer the doubts of the patient and family members, tell the successful case of the operation, increase the patient's cognition of treatment, eliminate the nervousness of patients, and encourage patients to increase their confidence in overcoming the epidemic. It is also necessary to carefully check the instruments and equipment used in the operation in advance. Blood routine, electrocardiogram, liver function, kidney function, and other examinations were performed, and the patient was instructed to abstain from drinking, fasting, and rest as soon as possible with 8 h before surgery. (2) Intraoperative care: gauze rolls, tongue depressors, and mouthpieces at the bedside were prepared to prevent the risk of tongue biting during seizures. When the seizure occurs, the patient needs to be taken the occipital supine position, tilted head to one side, given oxygen support, and wrapped the tongue depressors with gauze and put it into the mouth between molars to prevent the false bite when spasm [9]. The nursing staff cooperates with the anaesthetist for intubation and indwelling catheters, protects the eyes and ear canal of the patient, and cooperates with the surgeon in the future to ensure the smooth progress of the operation. (3) Postoperative care: after operation, the nursing staff should do preventive and control work in advance and instruct the patient to take medication on time. When seizures occur, sedatives are injected, and the number and frequency of seizures are recorded. According to the patient's age, physical fitness, and daily habits, appropriate exercise prescriptions was formulated (such as aerobic exercise includes walking and so on). During exercise, it is better to feel warm all over and sweat slightly. In the process of exercise, you must always follow the gradual and orderly progress, do what you can, and persevere. Nursing staffs pay close attention to the patient's condition and mood, communicate with the patient more, play their favorite music, and guide the family members to carry out some routine care. When discharged, nursing staff told patients to eat light and easy to digest food, avoid eating spicy and stimulating food, develop good habits of work and rest, and quit smoking and alcohol.

#### 2.2.3. Clinical Evaluation

*(1) The patient's EEG image was observed to analyze the type of lesion*. 

*(2) The Bad Mood of the Two Groups Was Compared*. Anxiety and depression were assessed by self-rating anxiety scale (SAS) and self-rating depression scale (SDS) [10] at T0 (the morning of the next day after admission), T3 (the seventh day after surgery), and T4 (the morning before discharge), respectively. More than 50 points indicate the existence of anxiety and depression, and the higher the score is, the more serious the anxiety and depression.

*(3) The Nursing Satisfaction and Pain Degree of the Two Groups Were Compared*. The self-made satisfaction questionnaire was used to investigate the nursing satisfaction of the two groups, including the appearance, nursing attitude, nursing operation proficiency, and language in the nursing process. The total score is 100, >90 is very satisfied, 80–89 is basically satisfied, and <79 is dissatisfied. Satisfaction = (number of very satisfied cases + number of basic satisfaction cases)/total number of cases × 100%. The changes of body pain degree were compared at T0, T1 (the morning of the day before surgery), T2 (the end of surgery), T3, and T4. A visual analogue scale (VAS) score is used [11], with a total of 0–10 points, 0 is painless and 10 is severe pain. The higher the score, the more severe the pain.

*(4) The Stress Response of the Two Groups Was Compared*. A multiparameter monitor was used to detect the patient's heart rate (HR), systolic blood pressure (SBP), and diastolic blood pressure (DBP) at T0, T1, T2, and T3.

*(5) The Quality of Life of the Two Groups Was Compared*. The European Organization for Research and Treatment of Cancer Quality of Life Questionnaire-Core 30 (EORTC QLQ-30) [12] was used at T0 and T4 to assess the quality of life of patients, including physical function, social function, role function, cognitive function, and emotional function five areas. The full score of each indicator is 100 points; the higher the score, the higher the quality of life.

*(6) The Occurrence of Complications and Recurrence of Epilepsy Were Compared between the Two Groups*. Complications include hydrocephalus, cerebral hemorrhage, infection, and suffocation. The patient was followed up for one year after discharge, and the patient's recurrence was recorded.

#### 2.2.4. Statistical Analysis

SPSS 20.0 statistical software was used for data analysis. Measurement data were expressed as *x* *±* *s*, and the *t*-test was performed. Count data were expressed as rate, and the *χ*^2^ test was performed. *P* < 0.05 indicates that the difference is statistically significant.

## 3. Results

### 3.1. EEG Test Results

During the surgery, 86 patients with epilepsy brain tumors were found to have spikes in 35 cases (7 meningiomas, 22 gliomas, and 6 cholesteatomas), 27 cases of sharp waves (14 meningiomas, 12 gliomas, and 1 case of cholesteatomas), and 24 cases of complex wave (9 cases of meningioma, 13 cases of glioma, and 2 cases of cholesteatoma) (Figure 1).

### 3.2. Comparison of SAS and SDS Scores between the Two Groups

There was no statistically significant difference in the SAS and SDS scores between the two groups at T0 (*P* > 0.05) (Figure 2). At T3 and T4, the SAS and SDS scores of the two groups decreased compared with T0, especially in the observation group (*P* < 0.05) (Figure 2).

### 3.3. Comparison of Pain Degree and Nursing Satisfaction between the Two Groups

The nursing satisfaction of the observation group (93.02%) was higher than that in the control group (79.07%) (*P* < 0.05) (Table 2). There was no significant difference in the VAS score between the two groups at T0 (*P* > 0.05) (Figure 3). The VAS score increased at T1 and T2, but decreased at T3 and T4, and the increase/decrease of the observation group was greater than that of the control group (*P* < 0.05) (Figure 3).

### 3.4. Comparison of Stress Response between the Two Groups

There was no significant difference in HR, SBP, and DBP between the two groups at T0 (*P* > 0.05) (Figure 4). At T1 and T2, the three indicators of the two groups all showed an upward trend, but they all decreased at T3, and the observation group increased/declined more significantly than the control group (*P* < 0.05) (Figure 4).

### 3.5. Comparison of the Quality of Life between the Two Groups

There was no statistically significant difference in the scores of the quality of life indicators between the two groups at T0 (*P* > 0.05) (Table 3). At T4, the scores of the quality of life indicators in the two groups increased, and the observation group increased more significantly than the control group (*P* < 0.05) (Table 3).

### 3.6. Comparison of Complication Rate and Recurrence Rate between the Two Groups

The complication rate and recurrence rate of the observation group were 4.65% and 2.33% and the control group were 23.26% and 13.95% (Table 4). The difference between the two groups was statistically significant (*P* < 0.05) (Table 4).

## 4. Discussion

Epilepsy is a common clinical symptom in patients with brain tumors, mostly in people between 20 and 60 years old [13, 14]. The occurrence of the symptom is due to the continuous growth of the lesion tissue in the brain that will cause compression and stimulation to the brain nerve, and the disease will appear with insufficient blood supply, hypoxia, brain edema, and so on with the progress, thus inducing epilepsy symptoms [15]. Therefore, the removal of epileptic foci is the main measure to treat brain tumors complicated by epilepsy. At present, the main clinical treatment for brain tumors is surgical resection [16]. With the improvement of medical concepts, the use of cortical EEG in monitoring and removing tumor and epileptic waves has been gradually applied in clinical practice. Its advantage is that those lesion complexes that cannot be observed in the naked eye can be removed under the guidance of cortical electrode, thus avoiding intraoperative residual lesions, effectively preventing postoperative intractable epilepsy, and greatly improving the clinical cure rate [17–20]. According to reports, patients with brain tumors have the highest incidence of epilepsy in patients with teratomas and lipomas, followed by oligodendroglioma, meningioma, poorly differentiated astrocytoma, cavernous hemangioma, and cholesteatoma [21, 22]. The majority of cases in this study were glioma and meningioma, which is consistent with previous study [21, 22]. A number of studies have shown that patients with brain tumors need to bear great mental pressure, combined with the trauma caused by surgical treatment to the body, will produce stress response, so that patients with brain tumors accompanied by epilepsy are easy to relapse after surgery [23–25]. Therefore, the implementation of scientific and comprehensive nursing intervention is particularly important.

This study adopts perioperative comprehensive nursing, which can start from the patients' physiology, psychology, treatment, recovery, and other aspects. Comprehensive intervention was carried out in the three stages of preoperative, operative, and postoperative, respectively, so as to meet the patients' physiological health needs, eliminate their doubts, and enhance their treatment confidence. The results of this study showed that the SAS, SDS scores, nursing satisfaction, and quality of life in the observation group were higher than those in the control group. The pain degree, stress response, complication rate, and recurrence rate in the observation group were lower than those in the control group. It is suggested that the perioperative comprehensive nursing intervention for patients with brain tumor accompanied with epilepsy who underwent operation under cortical EEG monitoring can eliminate the adverse psychological mood of patients, improve nursing satisfaction and quality of life, and reduce the degree of pain and stress response of patients, thus avoiding and reducing the occurrence of complications and recurrence. In this study, comprehensive perioperative nursing intervention was implemented for patients in the observation group. Before the operation, we visited the patient to understand the patient's individualized symptoms, so as to better choose the appropriate treatment plan. In addition, adequate preparations and careful examinations were carried out before the operation, and psychological interventions were carried out to eliminate the patients' anxiety and depression and other unhealthy emotions, establish the patient's treatment confidence, and help improve the patient's treatment compliance, thereby enhancing the treatment effect. The adequate preparation before surgery enables the nurses in the operating room to fully understand the surgical procedures and habits of doctors and also master the use of various instruments. They can calmly respond to the emergency situations of patients during surgery, which is conducive to the smooth operation and success of surgery. After operation, the patient is instructed to take medication on time, pay attention to physical exercise and diet management, take care of complications, and closely observe the patient's condition to avoid recurrence of epilepsy.

## 5. Conclusions

In summary, the perioperative use of comprehensive nursing intervention for patients with brain tumors and epilepsy undergoing resection under the monitoring of cortical EEG can improve the effectiveness and safety of the treatment.

## Figures and Tables

**Figure 1:** Results of EEG examination.

**Figure 2:** Comparison of SAS and SDS scores between the two groups. (a) The comparison of SAS scores at T0, T3, and T4. (b) The comparison of SDS scores at T0, T3, and T4.

**Figure 3:** Comparison of pain levels between the two groups at T0–T4.

**Figure 4:** Comparison of stress response between the two groups. (a) The comparison of HR between the two groups at T0–T3. (b) The comparison of SBP between the two groups at T0–T3. (c) The comparison of DBP between the two groups at T0–T3.

**Table 1:** Comparison of clinical data between the two groups (*n*).

Indicators	Observation	Control	*χ* ^2^	*P*
Cases	43	43		
Gender			0.195	>0.05
** **Male	27	25		
** **Female	16	18		
Age (years)			0.198	>0.05
** **>45	22	24		
** **≤45	21	19		
Position of the tumor			0.510	>0.05
** **Temporal lobe	10	11		
** **Frontal lobe	16	18		
** **Parietal lobe	9	8		
** **Occipital lobe	8	6		
Seizure type			0.190	>0.05
** **Generalized seizures	13	12		
** **Partial seizures	21	23		
** **Psychomotor seizures	9	8		
Pathological type			0.436	>0.05
** **Meningiomas	14	16		
** **Gliomas	25	22		
** **Cholesteatomas	4	5		

**Table 2:** Comparison of nursing satisfaction between the two groups (*n* (%)).

Group	*n*	Very satisfied	Basically satisfied	Dissatisfied	Satisfaction
Observation	43	23 (53.49)	17 (39.53)	3 (6.98)	40 (93.02)
Control	43	13 (30.23)	21 (48.84)	9 (20.93)	34 (79.07)
*χ* ^2^					6.199
*P*					<0.05

**Table 3:** Comparison of quality of life between the two groups ($\overset{-}{x}$ ± *s*).

Indicators	Time	Observation	Control	*t*	*P*
*N*		43	43		

Physical function	T0	62.33 ± 6.37	62.46 ± 6.23	0.284	>0.05
	T4	87.52 ± 6.74	75.67 ± 6.81	6.751	<0.05

Role function	T0	64.92 ± 7.84	65.38 ± 7.42	1.362	>0.05
	T4	90.23 ± 6.15	75.87 ± 6.62	7.753	<0.05

Emotional function	T0	61.19 ± 6.27	61.45 ± 6.68	0.582	>0.05
	T4	88.32 ± 7.14	75.62 ± 6.28	7.420	<0.05

Cognitive function	T0	65.12 ± 5.54	65.35 ± 5.27	0.158	>0.05
	T4	89.68 ± 7.85	78.63 ± 6.64	10.337	<0.05

Social function	T0	62.02 ± 5.56	62.73 ± 5.41	0.396	>0.05
	T4	87.93 ± 6.82	74.64 ± 6.47	4.785	<0.05

T0 is the morning after admission. T4 is the morning before discharge.

**Table 4:** Comparison of complication rate and recurrence rate between the two groups (*n* (%)).

Group	*n*	Hydrocephalus	Cerebral hemorrhage	Infection	Asphyxy	Incidence rate	Recurrence rate
Observation	43	1	0	1	0	2 (4.65)	1 (2.33)
Control	43	5	1	3	1	10 (23.26)	6 (13.95)
*χ* ^2^						10.623	4.530
*P*						<0.05	<0.05

## Data Availability

The data used to support the findings of this study are available from the corresponding author upon request.
